The article "Statistical Analysis of the People Fully Vaccinated against COVID-19 in Two Different Regions" was retracted in 2023. Reasons: signs of a paper mill; compromised peer review; unreliable results or conclusions.

# Statistical Analysis of the People Fully Vaccinated against COVID-19 in Two Different Regions

**DOI:** 10.1155/2022/7104960

**Published:** 2022-02-23

**Authors:** Abdullah Ali H. Ahmadini, Mohammed Elgarhy, A. W. Shawki, Hanan Baaqeel, Omar Bazighifan

**Affiliations:** ^1^Department of Mathematics, Faculty of Science, Jazan University, Jazan, Saudi Arabia; ^2^The Higher Institute of Commercial Sciences, Al Mahalla Al Kubra, 31951, Algarbia, Egypt; ^3^Central Agency for Public Mobilization & Statistics (CAPMAS), Cairo, Egypt; ^4^Statistics Department, Faculty of Science, King Abdulaziz University, Jeddah, Saudi Arabia; ^5^Department of Mathematics, Faculty of Science, Hadhramout University, Hadhramout 50512, Yemen

## Abstract

*Motivation*. Currently, the COVID-19 pandemic represents a critical issue all over the world. On May 11, 2020, at 05 : 41 GMT, approximately 0.28 million individuals had perished because of the COVID-19 pandemic, and the figure is continuously growing rapidly. Unfortunately, millions of people have died due to this pandemic. As a result, this issue forced governments and other corresponding organizations to take significant action, such as the lockdown and vaccinations. Furthermore, scientists have developed several vaccinations, and the World Health Organization (WHO) has urged governments and people to get vaccinated to eradicate this pandemic. Consequently, the findings of any scientific research into this phenomenon are highly interesting. *Problem Statement*. To enhance individual protection, it is now critical to analyze and compare the percentage of people fully vaccinated against COVID-19. It is constantly of interest in the field of big data science and other related disciplines to provide the best analysis and modeling of COVID-19 data. *Methodology*. Through this paper, we aimed to compare individuals who have been completely vaccinated against COVID-19 in two locations: North American countries and Arabian Peninsula countries. Simple techniques for comparing individuals who have been completely vaccinated against COVID-19 have been applied, which may be used to generate the foundation for conclusions. Most significantly, a modern statistical model was created to present the best assessment of individuals completely vaccinated against COVID-19 data in nations in North America and the Arabian Peninsula. Some of the suggested statistical model features were proposed. Furthermore, the estimate of the model parameters was driven using the maximum likelihood estimation method. *Results*. The flexibility provided by the proposed statistical model is useful for describing the percentage of the individuals completely vaccinated against COVID-19, which provides a close fit with the COVID-19 data. *Implications*. The proposed statistical model can be used for statistics and generate new statistical distributions that can be used to compare and predict the process of people's willingness to vaccinate and take the vaccine to try to eliminate COVID-19.

The article "Statistical Analysis of the People Fully Vaccinated against COVID-19 in Two Different Regions" was retracted in 2023. Reasons: signs of a paper mill; compromised peer review; unreliable results or conclusions.

## 1. Introduction

The first COVID-19 infection was discovered in the Chinese city of Wuhan, which is home to a well-known seafood wholesale market. The Wuhan Municipal Health Commission produced a total of 27 pneumonia cases of unknown origin on December 31, 2019. According to preliminary findings, the people involved with the wholesale company were originally infected with SARS and MERS via zoonotic transmission (the transmission of illness from an animal to a human). This infection spread rapidly and infected the entire city. More information about the pandemic can be found at https://en.wikipedia.org/wiki/Coronavirus_disease_2019. The examination of COVID-19 epidemic patterns across nations is quite concerning. In this connection, academics are making their best attempts to develop a strategy that will aid in the containment of this worldwide epidemic. Earlier attempts to compare epidemic dynamics in Italy and mainland China were described; see [1, 2] for more information. Reference [3] provides a comparison of the epidemic dynamics in Ukraine and surrounding nations. The COVID-19 is compared in Europe, the United States, and South Korea in reference [4]. We suggest interested readers to go to [5–19] for further information.

The World Health Organization (WHO) has been keen to urge governments and people to take the vaccine, in order to eliminate the pandemic and reduce the increasing number of deaths and injuries.

In the present circumstances, it is of tremendous interest to learn more about people who have been completely vaccinated against COVID-19 and to compare as many different nations as appropriate. As a result, an attempt has been made in this article to compare the people fully vaccinated against COVID-19, in the two distinct areas of North America and the Arabian Peninsula.

This article is sorted into sections: Section 2 compares people who have been completely immunized against COVID-19 in two distinct regions: North America and the Arabian Peninsula.  Section 3 describes the suggested statistical model.  Section 4 describes some of the suggested statistical model's features. The estimate of the model parameters is presented in Section 5. Parameter estimation by the maximum likelihood estimation method is discussed in Section 6.  Section 7 is focused on the simulation of COVID-19 occurrences. Eventually, the article is concluded in the last part.

The article "Statistical Analysis of the People Fully Vaccinated against COVID-19 in Two Different Regions" was retracted in 2023. Reasons: signs of a paper mill; compromised peer review; unreliable results or conclusions.

## 2. Comparison of People Fully Vaccinated against COVID-19 in Different Regions

In this section, we will look at a quick and easy way to compare people who have been fully vaccinated against COVID-19 in two different parts of the world: North America and the Arabian Peninsula. The comparison is made by considering the percentage of people fully vaccinated against COVID-19. The comparison of the percentage of people fully vaccinated against COVID-19 in North American countries and Arabian Peninsula countries is presented in Tables 1 and 2, as well as in Figures 1 and 2.

## 3. The Proposed Statistical Model

There has been a growing interest in establishing new statistical models or new families of statistical models in the practice of big data sciences, particularly in statistical theory, to offer a clearer explanation of the problems under discussion.

Adding new parameter(s) to a class of distribution functions often offers them greater flexibility, enhances their features, and provides better fits to real-world data than other modified models. However, on the other side, there is an issue with parametrization. We extend this field of statistical theory and offer a new statistical model to avoid such difficulties and provide a better representation of real-world occurrences. The proposed distribution may be called the double weighted quasi Lindley (DWQL) distribution.

Reference [20] studied quasi Lindley (QL) distribution, and it has the following pdf as

(1) $$\begin{array}{c} f\left(x,\alpha ,\theta \right)=\frac{\theta }{1+\alpha }\left(\alpha +\theta x\right)e^{-\theta x};x>0,\theta >0,\alpha >‐1. \end{array}$$

When *α* = *θ*, we can get the Lindley (*L*) distribution which studied by [21].

Reference [22] suggested the pdf of double weighted models as

(2) $$\begin{array}{c} f_{w}\left(x\right)=\frac{w\left(x\right)f\left(x\right)F\left(x\right)}{W_{D}},x\geq 0, \end{array}$$

where

(3) $$\begin{array}{c} W_{D}=\int_{0}^{\infty }w\left(x\right)f\left(x\right)F\left(x\right)\;dx. \end{array}$$

Using (1) in (2) and let *w*(*x*) = *x*, the pdf of the model is

(4) $$\begin{array}{c} f_{\text{DWQL}}\left(x,\alpha ,\theta \right)=\frac{\theta^{3}\left(\alpha x^{2}+\theta x^{3}\right)}{2\left(\alpha +3\right)}e^{-\theta x},x\geq 0,\theta ,\alpha >0. \end{array}$$

The distribution function (cdf), the reliability (*R*), and the hazard rate (hr) functions are given by

(5) $$\begin{array}{c} F_{\text{DWQL}}\left(x,\alpha ,\theta \right)=1-\left[1+\theta x+\frac{\theta^{2}x^{2}}{2}+\frac{\theta^{3}x^{3}}{2\left(\alpha +3\right)}\right]e^{-\theta x}, \end{array}$$

(6) $$\begin{array}{c} R\left(x,\alpha ,\theta \right)=\bar{F}\left(x,\alpha ,\theta \right)=\left[1+\theta x+\frac{\theta^{2}x^{2}}{2}+\frac{\theta^{3}x^{3}}{2\left(\alpha +3\right)}\right]e^{-\theta x}, \end{array}$$

(7) $$\begin{array}{c} h\left(x,\alpha ,\theta \right)=\frac{f\left(x,\alpha ,\theta \right)}{\bar{F}\left(x,\alpha ,\theta \right)}=\frac{\theta^{3}\left(\alpha x^{2}+\theta x^{3}\right)}{2\left(\alpha +3\right)\left[1+\theta x+\left(\theta^{2}x^{2}/2\right)+\left(\theta^{3}x^{3}/2\left(\alpha +3\right)\right)\right]}. \end{array}$$

Figures 3–6 provide the pdf, cdf, R, and the hr functions of DWQL model.

The article "Statistical Analysis of the People Fully Vaccinated against COVID-19 in Two Different Regions" was retracted in 2023. Reasons: signs of a paper mill; compromised peer review; unreliable results or conclusions.

The DWQL is a very flexible model. The DWQL distribution contains special models according to its parameter values as follows:

1. If *α* = *θ*, then cdf (5) gives DWL (new)
2. If *α* = 0, we get the double *W* gamma (2, *θ*) model (new)

## 4. The Statistical Properties of DWQLD

The *r*th moment of *X* is supplied via

(8) μr′=ΕXr=∫0∞xrfDWQLx,α,θdx=θ32α+3α∫0∞xr+2e−θxdx+θ∫0∞xr+3e−θxdx=θ32α+3αr+3θr+3+θr+4θr+4,μr′=r+32α+3θrα+r+3.

The mean *E*(*X*), variance (var), and coefficient of variation of this distribution are

(9) $$\begin{array}{c} E\left(X\right)=\mu_{1}^{\prime }\left(x\right)=\frac{2\left(\alpha +3\right)}{\left(\alpha +2\right)\theta },\\ \mathrm{var}=E\left(X^{2}\right)‐{\left[E\left(X\right)\right]}^{2}=\frac{3\left(\alpha^{2}+8\alpha +12\right)}{{\left(\alpha +3\right)}^{2}\theta^{2}},\\ \text{CV}=\frac{\sigma }{\mu }=\frac{{\left(3\alpha^{2}+24\alpha +36\right)}^{1/2}}{2\theta {\left(\alpha +3\right)}^{2}}. \end{array}$$

Some numerical values of moments are presented in Tables 3–6.

From the previous tables, we can note the following:

- In Tables 3 and 4, when the value of *α* is increasing, then the values of *E*(*X*), *E*(*X*^2^), *E*(*X*^3^), *E*(*X*^4^), and var are decreasing while the values of CV are increasing
- In Tables 5 and 6, when the value of *α* is increasing, then the values of *E*(*X*), *E*(*X*^2^), *E*(*X*^3^), *E*(*X*^4^), and var are decreasing while the values of CV are constant

The moment generating function *M*_*X*_(*t*) has the following form:

(10) $$\begin{array}{c} {Μ}_{X}\left(t\right)=E\left(e^{tX}\right)=\int_{0}^{\infty }e^{tx}f_{\text{DWQL}}\left(x,\alpha ,\theta \right)\;dx=\int_{0}^{\infty }e^{tx}\frac{\theta^{3}\left(\alpha x^{2}+\theta x^{3}\right)}{2\left(\alpha +3\right)}e^{-\theta x}\;dx=\frac{\theta^{3}}{\left(\alpha +3\right)}\left[\frac{\alpha }{{\left(\theta -t\right)}^{3}}+\frac{3\theta }{{\left(\theta -t\right)}^{4}}\right]. \end{array}$$

Let *X*_1:*n*_ < *X*_2:*n*_ < , ⋯, <*X*_*n*:*n*_ denote the order statistics taken from this sample. The pdf of the *j*th order statistic, say *f*_*j*:*n*_(*x*, *φ*), is

(11) $$\begin{array}{c} f_{j:n}\left(x,\Phi \right)=\frac{1}{B\left(j,n-j+1\right)}{\left[F\left(x,\varphi \right)\right]}^{j-1}{\left[1-F\left(x,\varphi \right)\right]}^{n-j}f\left(x,\varphi \right), \end{array}$$

Inserting (4) and (5) into (11), we get the pdf of the *j*th order statistic as follows:

(12) $$\begin{array}{c} f_{X_{\left(j\right)}}\left(x\right)=\frac{n!}{\left(j-1\right)!\left(n-j\right)!}f\left(x\right){\left[F_{\left(x\right)}\right]}^{j-1}{\left[1-F_{\left(x\right)}\right]}^{n-j}=\frac{n!}{\left(j-1\right)!\left(n-j\right)!}\frac{\theta^{3}x^{2}\left(\alpha +\theta x\right)e^{-\left(n-j+1\right)\theta x}}{2\left(\alpha +3\right)}{\left[1+\theta x+\frac{\theta^{2}x^{2}}{2}+\frac{\theta^{3}x^{2}}{2\left(\alpha +3\right)}\right]}^{n-j}\times {\left[1-\left[1+\theta x+\frac{\theta^{2}x^{2}}{2}+\frac{\theta^{3}x^{2}}{2\left(\alpha +3\right)}\right]e^{-\theta x}\right]}^{j-1}. \end{array}$$

The pdf *f*_*X*_(1)__(*x*) of the first order statistic is given by

(13) $$\begin{array}{c} f_{X_{\left(1\right)}}\left(x\right)=n{\left[1-F_{\left(x\right)}\right]}^{n-1}f_{\left(x\right)}=\frac{n\;\theta^{3}x^{2}\left(\alpha +\theta x\right)e^{-n\theta x}\;}{2\left(\alpha +3\right)}{\left[1+\theta x+\frac{\theta^{2}x^{2}}{2}+\frac{\theta^{3}x^{3}}{2\left(\alpha +3\right)}\right]}^{n-1}. \end{array}$$

The pdf *f*_*X*_(*n*)__(*x*) of the largest order statistic is given by

(14) $$\begin{array}{c} f_{X_{\left(n\right)}}\left(x\right)=n{\left[F_{\left(x\right)}\right]}^{n-1}f_{\left(x\right)}=\frac{n\;\theta^{3}x^{2}\left(\alpha +\theta x\right)e^{-\theta x}\;}{2\left(\alpha +3\right)}{\left\{1-\left[1+\theta x+\frac{\theta^{2}x^{2}}{2}+\frac{\theta^{3}x^{3}}{2\left(\alpha +3\right)}\right]e^{-\theta x}\right\}}^{n-1}. \end{array}$$

The joint pdf of *x*_*j*_ and *x*_*k*_ (for *x*_*j*_ < *x*_*k*_) is given by

(15) $$\begin{array}{c} f_{X_{j}.X_{k}\left(x_{j}.x_{k}\right)}=\frac{n!}{\left(j-1\right)!\left(k-j-1\right)!\left(n-k\right)!}{\left[F\left(x_{j}\right)\right]}^{j-1}{\left[F\left(x_{k}\right)-F\left(x_{j}\right)\right]}^{k-j-1}{\left[1-F\left(x_{k}\right)\right]}^{n-k}f\left(x_{j}\right).f\left(x_{k}\right)=\frac{n!}{\left(j-1\right)!\left(k-j-1\right)!\left(n-k\right)!}\frac{\;2\theta^{3}x_{j}^{2}x_{k}^{2}\left(\alpha +\theta x_{j}\right)\left(\alpha +\theta x_{k}\right)e^{-\theta x_{j}}e^{-\left(1+n-k\right)\theta x_{k}}\;}{4\left(\alpha +3\right)}\times {\left\{1-\left[1+\theta x_{j}+\frac{\theta^{2}x_{j}^{2}}{2}+\frac{\theta^{3}x_{j}^{3}}{2\left(\alpha +3\right)}\right]e^{-\theta x_{j}}\right\}}^{j-1}{\left[1+\theta x+\frac{\theta^{2}x_{k}^{2}}{2}+\frac{\theta^{3}x_{j}^{3}}{2\left(\alpha +3\right)}\right]}^{n-k}\times {\left\{\left[1-\left[1+\theta x+\frac{\theta^{2}x_{k}^{2}}{2}+\frac{\theta^{3}x_{k}^{3}}{2\left(\alpha +3\right)}\right]e^{-\theta x_{k}}\right]-\left[1-\left[1+\theta x_{j}+\frac{\theta^{2}x_{j}^{2}}{2}+\frac{\theta^{3}x_{j}^{3}}{2\left(\alpha +3\right)}\right]e^{-\theta x_{j}}\right]\right\}}^{k-j-1}. \end{array}$$

The article "Statistical Analysis of the People Fully Vaccinated against COVID-19 in Two Different Regions" was retracted in 2023. Reasons: signs of a paper mill; compromised peer review; unreliable results or conclusions.

## 5. Maximum Likelihood

Let *X*_1_, X_2_, ⋯, *X*_*n*_ be a random sample of size *n* from DWQL(*x*, *ϕ*). Taking the log-likelihood function for the vector of parameters *ϕ* = (*α*, *θ*), we get

(16) $$\begin{array}{c} \log\;L=‐n\;\log\;2+3n\;\log\;\theta ‐n\;\log\;\left(\alpha +3\right)+\overset{n}{\underset{i=1}{\sum }}\log\;{x_{i}}^{2}‐\theta \overset{n}{\underset{i=1}{\sum }}x_{i}+\overset{n}{\underset{i=1}{\sum }}\log\left(\alpha +\theta x_{i}\right). \end{array}$$

The score vector's components are given by

(17) $$\begin{array}{c} \frac{\partial \log L}{\partial \theta }=\frac{3n}{\theta }-\overset{n}{\underset{i=1}{\sum }}x_{i}+\overset{n}{\underset{i=1}{\sum }}\frac{x_{i}}{\alpha +\theta x_{i}}, \end{array}$$

(18) $$\begin{array}{c} \frac{\partial \log L}{\partial \alpha }=\frac{-n}{\alpha +3}+\overset{n}{\underset{i=1}{\sum }}\frac{1}{\alpha +\theta x_{i}}. \end{array}$$

Set these nonlinear equations (17) and (18) to zero and solve them concurrently to get estimates of the unknown values of parameters *α* and *θ*. The second partial derivatives of *L* are

(19) $$\begin{array}{c} \frac{\partial \log L}{\partial \theta^{2}}=-\frac{3n}{\theta^{2}}-\overset{n}{\underset{i=1}{\sum }}\frac{x_{i}^{2}}{{\left(\alpha +\theta x_{i}\right)}^{2}},\\ \frac{\partial \log L}{\partial \alpha^{2}}=\frac{n}{{\left(\alpha +3\right)}^{2}}-\overset{n}{\underset{i=1}{\sum }}\frac{1}{{\left(\alpha +\theta x_{i}\right)}^{2}},\\ \frac{\partial \log L}{\partial \theta \;\partial \alpha }=\overset{n}{\underset{i=1}{\sum }}\frac{x_{i}}{{\left(\alpha +\theta x_{i}\right)}^{2}}, \end{array}$$

where

(20) $$\begin{array}{c} V_{\alpha \alpha }=\frac{\partial^{2}\log L}{\partial \alpha^{2}},\\ V_{\theta \theta }=\frac{\partial^{2}\log L}{\partial \theta^{2}},\\ V_{\alpha \theta }=\frac{\partial^{2}\log L}{\partial \alpha \partial \theta }. \end{array}$$

## 6. Numerical Outcomes

In this part, we evaluate the ML estimators' performance in terms of sample size *n*. A numerical evaluation of the performance of ML estimators for the DWQL distribution is performed. Estimates are *X*_1_, *X*_2_, ⋯, *X*_*n*_ evaluated using the Mathematica program based on the following quantities for each sample size: empirical mean square errors (MSEs). The following are the numerical procedures:

- A random sample of sizes *n* = 30, 50, 100, 200, and 300 is taken into account; these random samples are produced from the DWQL distribution using the inversion approach
- Four sets of parameters are taken into account
- The DWQL model's ML estimates (MLEs) are assessed for each parameter value and sample size
- Repeat this process 10000 times to obtain the means and MSEs of the MLE for various parameter values in both models and for each sample size
- Tables 7 and 8 present empirical findings. These tables show that the estimates are fairly consistent and near to the real value of the parameters as sample sizes grow

The article "Statistical Analysis of the People Fully Vaccinated against COVID-19 in Two Different Regions" was retracted in 2023. Reasons: signs of a paper mill; compromised peer review; unreliable results or conclusions.

## 7. Modelling to the People Fully Vaccinated against COVID-19

This section concerned with two important real data sets. The first data called the percentage of people fully vaccinated against COVID-19 in North American countries to 6 Oct 2021. The dataset was obtained from the following electronic address: https://ourworldindata.org/covid-vaccinations?country=OWID_WRL. The data set is reported in Table 1.

The second data represent the percentage of the share of people fully vaccinated against COVID-19 in the Arabian Peninsula countries to 6 Oct 2021. The dataset was obtained from the following electronic address: https://ourworldindata.org/covid-vaccinations?country=OWID_WRL. The data set is reported in Table 2. The descriptive analysis of the both data sets is reported in Tables 9 and 10.

In this section, two above data sets are studied to show how the DWQL distribution outperforms other models. Comparing the new model to some models, namely, exponential Poisson Lindley (EPL), extended generalized Lindley (EGL), extended Lindley (EL), generalized inverse Lindley (GIL), and the odd Burr Lindley (OBL) models, we obtain the MLEs and standard errors (SEs) of the model parameters. To compare the distribution models, we consider criteria like Akaike information criterion (AIC), the correct AIC (CAIC), Bayesian IC (BIC), Hannan-Quinn IC (HQIC), Kolmogorov–Smirnov (KS) test, and *p* value (PV) test. The wider distribution, on the other hand, refers to lower AIC, CAIC, BIC, HQIC, KS, and the greatest value of PV.

The MLEs of the six competitive models and their SEs and values of AIC, CAIC, BIC, HQIC, PV, and KS for the both data sets are presented in Tables 11 and 12.

We find that the DWQL distribution with two parameters provides a better fit than five models. It has the smallest values of AIC, CAIC, BIC, HQIC, and KS and the greatest value of PV among those considered here.

Moreover, the plots of empirical cdf, empirical pdf, and PP plots of our competitive model for the both data sets are displayed in Figures 7–10, respectively.

The DWQL model clearly gives the best overall fit and so may be picked as the most appropriate model for explaining data.

The article "Statistical Analysis of the People Fully Vaccinated against COVID-19 in Two Different Regions" was retracted in 2023. Reasons: signs of a paper mill; compromised peer review; unreliable results or conclusions.

## 8. Summary and Conclusion

COVID-19 is one of the most dangerous viruses that has had a significant impact on daily life. The government, as well as a number of other organizations, should really be capable of providing comparison bases and a clearer description of the data under examination in order to obtain credible estimates of the parameters of interest. A brief comparison of the COVID-19 events, such as a person fully vaccinated against COVID-19 in two different regions, is provided. Such a detailed comparison should aid in understanding the percentage of people completely vaccinated against COVID-19 in various nations. A novel statistical model is also introduced. The suggested model's mathematical characteristics are then deduced. The model parameters' maximum likelihood estimators are produced. Parameter estimation by the maximum likelihood estimation method is discussed. The flexibility provided by the proposed model could be very useful in adequately describing the percentage of people completely vaccinated against COVID-19 in different countries. We observed that the proposed model may provide a close fit to the percentage of people completely vaccinated against COVID-19 in different countries' data.

## Figures and Tables

**Figure 1:** Bar chart of percentage of person completely vaccinated against COVID-19 in North American countries.

**Figure 2:** Bar chart of percentage of person completely vaccinated against COVID-19 in the Arabian Peninsula countries.

**Figure 3:** The pdf of DWQL model.

**Figure 4:** The cdf of DWQL model.

**Figure 5:** The R function of DWQLD.

**Figure 6:** The hr function of DWQL model.

**Figure 7:** Estimated pdf and cdf of competitive model for the first data set.

**Figure 8:** PP plot of the fitted model for the first data set.

**Figure 9:** Estimated pdf and cdf of competitive model for the second data set.

**Figure 10:** PP plot of the fitted model for the first data set.

**Table 1:** In North American countries, the percentage of people who have been fully immunized against COVID-19.

Country	Fully vaccinated against %	Country	Fully vaccinated against %	Country	Fully vaccinated against %
Anguilla	0.6054	Cuba	0.4811	Mexico	0.3607
Antigua and Barbuda	0.4444	Curacao	0.5454	Montserrat	0.2787
Aruba	0.7044	Dominica	0.2988	Nicaragua	0.0455
Bahamas	0.2224	Dominican Republic	0.4516	Panama	0.5238
Barbados	0.3762	El Salvador	0.5437	Saint Kitts and Nevis	0.4187
Belize	0.3437	Greenland	0.6369	Saint Lucia	0.1888
Bermuda	0.6929	Grenada	0.2163	Saint Vincent and the Grenadines	0.1218
British Virgin Islands	0.5049	Guatemala	0.1463	Sint Maarten (Dutch part)	0.5486
Canada	0.7174	Haiti	0.002	Trinidad and Tobago	0.3785
Cayman Islands	0.8346	Honduras	0.2416	Turks and Caicos Islands	0.6355
Costa Rica	0.4457	Jamaica	0.0999	United States	0.5549

The article "Statistical Analysis of the People Fully Vaccinated against COVID-19 in Two Different Regions" was retracted in 2023. Reasons: signs of a paper mill; compromised peer review; unreliable results or conclusions.

**Table 2:** Percentage of person completely vaccinated against COVID-19 in the Arabian Peninsula countries.

Country	Completely vaccinated against %
Bahrain	0.6446
Iraq	0.0712
Jordan	0.3264
Oman	0.3926
Qatar	0.757
Saudi Arabia	0.5519
United Arab Emirates	0.8395

**Table 3:** Summary statistics of some moments of DWQL distribution at *θ* = 3.0 and various values of *α*.

*α*	*E*(*X*)	*E*(*X*^2^)	*E*(*X*^3^)	*E*(*X*^4^)	var	CV
0.200	1.313	2.167	4.306	10.000	0.444	0.508
0.400	1.294	2.118	4.183	9.673	0.443	0.514
0.800	1.278	2.074	4.074	9.383	0.441	0.520
1.000	1.263	2.035	3.977	9.123	0.440	0.525
1.200	1.250	2.000	3.889	8.889	0.438	0.529
1.400	1.238	1.968	3.810	8.677	0.435	0.533
1.600	1.227	1.939	3.737	8.485	0.433	0.536
1.800	1.217	1.913	3.672	8.309	0.431	0.539
2.000	1.208	1.889	3.611	8.148	0.429	0.542
2.200	1.200	1.867	3.556	8.000	0.427	0.544
2.400	1.192	1.846	3.504	7.863	0.425	0.547
2.600	1.185	1.827	3.457	7.737	0.423	0.548
2.800	1.179	1.810	3.413	7.619	0.421	0.550
3.000	1.172	1.793	3.372	7.510	0.419	0.552

**Table 4:** Summary statistics of some moments of DWQL distribution at *θ* = 5.0 and various values of *α*.

*α*	*E*(*X*)	*E*(*X*^2^)	*E*(*X*^3^)	*E*(*X*^4^)	var	CV
0.200	0.788	0.780	0.930	1.296	0.160	0.508
0.400	0.777	0.762	0.904	1.254	0.159	0.514
0.800	0.767	0.747	0.880	1.216	0.159	0.520
1.000	0.758	0.733	0.859	1.182	0.158	0.525
1.200	0.750	0.720	0.840	1.152	0.158	0.529
1.400	0.743	0.709	0.823	1.125	0.157	0.533
1.600	0.736	0.698	0.807	1.100	0.156	0.536
1.800	0.730	0.689	0.793	1.077	0.155	0.539
2.000	0.725	0.680	0.780	1.056	0.154	0.542
2.200	0.720	0.672	0.768	1.037	0.154	0.544
2.400	0.715	0.665	0.757	1.019	0.153	0.547
2.600	0.711	0.658	0.747	1.003	0.152	0.548
2.800	0.707	0.651	0.737	0.987	0.151	0.550
3.000	0.703	0.646	0.728	0.973	0.151	0.552

**Table 5:** Summary statistics of some moments of DWQL distribution at *α* = 5.0 and various values of *θ*.

*θ*	*E*(*X*)	*E*(*X*^2^)	*E*(*X*^3^)	*E*(*X*^4^)	var	CV
0.200	16.875	375.000	10312.500	337500.000	90.234	0.563
0.400	8.438	93.750	1289.063	21093.750	22.559	0.563
0.800	5.625	41.667	381.944	4166.667	10.026	0.563
1.000	4.219	23.438	161.133	1318.359	5.640	0.563
1.200	3.375	15.000	82.500	540.000	3.609	0.563
1.400	2.813	10.417	47.743	260.417	2.507	0.563
1.600	2.411	7.653	30.066	140.566	1.842	0.563
1.800	2.109	5.859	20.142	82.398	1.410	0.563
2.000	1.875	4.630	14.146	51.440	1.114	0.563
2.200	1.688	3.750	10.313	33.750	0.902	0.563
2.400	1.534	3.099	7.748	23.052	0.746	0.563
2.600	1.406	2.604	5.968	16.276	0.627	0.563
2.800	1.298	2.219	4.694	11.817	0.534	0.563
3.000	1.205	1.913	3.758	8.785	0.460	0.563

The article "Statistical Analysis of the People Fully Vaccinated against COVID-19 in Two Different Regions" was retracted in 2023. Reasons: signs of a paper mill; compromised peer review; unreliable results or conclusions.

**Table 6:** Summary statistics of some moments of DWQL distribution at *α* = 10 and various values of *θ*.

*θ*	*E*(*X*)	*E*(*X*^2^)	*E*(*X*^3^)	*E*(*X*^4^)	var	CV
0.200	16.154	346.154	9230.769	294230.800	85.207	0.571
0.400	8.077	86.539	1153.846	18389.420	21.302	0.571
0.800	5.385	38.462	341.880	3632.479	9.468	0.571
1.000	4.039	21.635	144.231	1149.339	5.325	0.571
1.200	3.231	13.846	73.846	470.769	3.408	0.571
1.400	2.692	9.615	42.735	227.030	2.367	0.571
1.600	2.308	7.064	26.912	122.545	1.739	0.571
1.800	2.019	5.409	18.029	71.834	1.331	0.571
2.000	1.795	4.274	12.662	44.845	1.052	0.571
2.200	1.615	3.462	9.231	29.423	0.852	0.571
2.400	1.469	2.861	6.935	20.096	0.704	0.571
2.600	1.346	2.404	5.342	14.189	0.592	0.571
2.800	1.243	2.048	4.202	10.302	0.504	0.571
3.000	1.154	1.766	3.364	7.659	0.435	0.571

**Table 7:** MLEs and MSE of DWQL distribution for set 1 and set 2.

*n*	Set 1 (0.5, 0.5)		Set 2 (0.5, 1.5)	
	MLE	MSE	MLE	MSE
30	0.519876	0.010675	0.549776	0.015231
	0.583619	0.096384	1.763210	0.652452
50	0.519020	0.006504	0.526846	0.006895
	0.580228	0.050699	1.731120	0.467523
100	0.507657	0.002476	0.512182	0.002960
	0.532262	0.013490	1.621920	0.109372
200	0.506596	0.001206	0.501286	0.001231
	0.504893	0.006243	1.561980	0.063621
300	0.503032	0.000785	0.501934	0.000863
	0.510978	0.003014	1.488500	0.028265

**Table 8:** MLEs and MSE of DWQL distribution for set 3 and set 4.

*n*	Set 3 (0.5, 2.0)		Set 4 (1.5, 1.5)	
	MLE	RMSE	MLE	RMSE
30	0.536645	0.013190	1.655650	0.215975
	2.312980	1.042390	1.658180	0.222000
50	0.514007	0.004442	1.597290	0.104171
	2.160900	0.424585	1.612420	0.106485
100	0.506586	0.003029	1.530670	0.035813
	2.009150	0.119023	1.519900	0.047282
200	0.502757	0.001286	1.508970	0.013951
	2.000800	0.090311	1.522580	0.019672
300	0.505382	0.000974	1.516210	0.013526
	2.071520	0.064444	1.523070	0.015873

**Table 9:** Some descriptive analysis of data set 1.

*n*	Mean	Median	*V*	SK	Range	Min	Max
33	0.412	0.444	0.045	-0.123	0.832	0.002	0.834

**Table 10:** Some descriptive analysis of data set 2.

*n*	Mean	Median	*V*	SK	Range	Min	Max
7	0.512	0.552	0.072	-0.504	0.768	0.071	0.840

**Table 11:** MLEs, SEs, and measures of fitting for the first data set.

Distributions	MLE and SE			AIC	CAIC	BIC	HQIC	KS	PV
	*β*	*α*	*θ*						
DWQL	8.196	4.884		9.399	9.799	8.436	10.406	0.13956	0.54136
	(1.528)	(11.389)							
EPL	2.424	1.886^∗^10^6^		11.549	11.949	10.586	12.556	0.23198	0.05735
	(5.896^∗^10^−8^)	(4.959^∗^10^11^)							
EGL	7.451	1.758	13.102	80.725	81.553	79.281	82.236	0.20803	0.11494
	(0.556)	(1.682)	(11.532)						
EL	1.468	11.212	0.273	14.638	15.466	13.194	16.149	0.22991	0.06108
	(0.703)	(9.198)	(0.282)						
GIL	0.7	0.48		56.171	56.571	55.208	57.178	0.32465	0.00191
	(0.116)	(0.047)							
OBL	0.229	0.954	11.85	13.08	13.908	11.636	14.591	0.23098	0.05912
	(0.07)	(0.109)	(8.738)						

The article "Statistical Analysis of the People Fully Vaccinated against COVID-19 in Two Different Regions" was retracted in 2023. Reasons: signs of a paper mill; compromised peer review; unreliable results or conclusions.

**Table 12:** The MLEs, SEs, and measures of fitting for the second data set.

Distributions	MLE and SE			AIC	CAIC	BIC	HQIC	KS	PV
	*β*	*α*	*θ*						
DWQL	5.862	3683		6.172	9.172	3.862	4.835	0.19871	0.94505
	(5.317^∗^10^−10^)	(2.965^∗^10^6^)							
EPL	1.954	5.239^∗^10^5^		8.625	11.625	6.315	7.288	0.48411	0.07518
	(1.81^∗^10^−8^)	(8.275^∗^10^10^)							
EGL	6.811	2.511	19.036	19.217	27.217	15.752	17.211	0.36247	0.31654
	(2.615)	(1.704)	(29.718)						
EL	1.232	3.258	3.397	7.511	15.511	4.046	5.505	0.39238	0.23133
	(0.642)	(8.359)	(5.307)						
GIL	0.558	0.875		11.483	14.483	9.174	10.146	0.29915	0.55806
	(0.227)	(0.207)							
OBL	0.147	1.603	9.126	10.264	18.264	6.799	8.259	0.32305	0.4582
	(1.007)	(0.19)	(6.835)						

## Data Availability

Please contact the relevant author if you would like to acquire the numerical dataset used to conduct the research described in the paper.
